The article "SAMMSON drives the self-renewal of liver tumor initiating cells through EZH2-dependent Wnt/β-catenin activation" was retracted in 2022. Reasons: duplicated images; original data or images not available.

# *SAMMSON* drives the self-renewal of liver tumor initiating cells through EZH2-dependent Wnt/β-catenin activation

**DOI:** 10.18632/oncotarget.21792

**Published:** 2017-10-10

**Authors:** Xiaopeng Li, Ming Li, JiaLi Chen, Hua Dai, Liang Wang, Ying Xiong, Yuanbin Zhong, Lunli Zhang

**Affiliations:** ^1^ Department of Infectious Disease, The First Affiliated Hospital of Nanchang University, Nanchang, JiangXi 330006, China; ^2^ Department of Function, JiangXi Children’s Hospital, Nanchang, JiangXi 330006, China; ^3^ Department of Pathology, The First Affiliated Hospital of Nanchang University, Nanchang, JiangXi 330006, China

**Keywords:** liver TICs, SAMMSON, EZH2, Wnt/β-catenin, self-renewal

## Abstract

Liver cancer is one of the most serious cancers all over the world. Liver tumor initiating cells (TICs) account for tumor initiation and metastasis. However, the regulatory mechanism of liver TICs remains unclear. Here we found long noncoding RNA *SAMMSON* is highly expressed in liver cancer and liver TICs. *SAMMSON* silenced cells show impaired self-renewal capacity, while, its overexpression induces enhanced self-renewal. *SAMMSON* drives the activation of Wnt/β-catenin signaling, and thus promotes liver TIC self-renewal. *SAMMSON* interacts with EZH2, a core component of PRC2 complex, and inhibits the expression of CTNNBIP1 through EZH2 dependent manner. *SAMMSON* binds to *CTNNBIP1* promoter and recruits EZH2 to *CTNNBIP1* promoter. What’s more, targeting liver TICs through *SAMMSON*, EZH2 and Wnt/β-catenin signaling impaired liver TIC self-renewal, decreased tumor propagation and severity. Taken together, *SAMMSON* drives liver TIC self-renewal through EZH2-dependent Wnt/β-catenin activation.

## INTRODUCTION

Liver cancer, including hepatocellular carcinoma (HCC) and cholangiocarcinoma, is one of the most serious cancers all over the world [1]; while, the mechanism of liver tumorigenesis is still unclear. Within several cell types in liver tumor bulk, a small subset of liver cancer cells, termed liver tumor initiating cells (TICs) are considered as the origin of liver cancer [2]. Liver TICs have the capacities of self-renewal and differentiation. They can repopulate themselves and generate all cell types in the tumor bulk [3]. According to the multiple characters of liver TICs, many experimental systems were developed. Sphere formation assay reflects the self-renewal of liver TICs [4]; side population assay mirrors the drug-resistance of liver TICs [5]; and gradient diluted xenograft assay detects the tumor initiating ability of liver TICs [6]. Along with the deep investigation on liver TICs, more and more surface markers have been discovered, including CD13, CD133, CD24, CD90 and so on [7–9]. Meanwhile, many signaling pathways participate in liver TICs. Wnt/β-catenin, Notch, Hedgehog and Hippo/Yap signaling pathways are most deeply investigated [10–12]. Recently, several transcription factors have been reported to participate in liver TIC self-renewal, including c-Myc, Oct4, Zic2, Sox4, Stat3 and so on [13, 14]. However, the biology and regulatory mechanism of liver TICs are still elusive.

The article "SAMMSON drives the self-renewal of liver tumor initiating cells through EZH2-dependent Wnt/β-catenin activation" was retracted in 2022. Reasons: duplicated images; original data or images not available.

Wnt/β-catenin signaling, one of the most important signaling in liver TICs, is regulated by many modulators [15]. The well-known regulatory mechanism is the switch between β-catenin disruption complex (APC complex) and stable complex (TCF/LEF complex)[16]. In Wnt-Off cells, APC complex disrupts β-catenin through β-TrCP induced ubiquitinoylation; while, in Wnt-On cells, APC complex was dissolved, followed by β-catenin nuclear translocation and activation through forming β-catenin-TCF/LEF complex [17]. CTNNBIP1, a physiological inhibitory protein of Wnt/β-catenin signaling, interacts with β-catenin and inhibits the interaction between β-catenin and TCF/LEF complex, and finally blocks the activation of Wnt/β-catenin signaling [18]. Although many molecules are involved in Wnt/β-catenin signaling, the role of lncRNAs in this progress is rarely reported.

Long noncoding RNAs (LncRNAs) are defined as RNA transcripts that contain more than 200 nucleotides in length without protein coding potential [19]. For long time, lncRNAs were considered as byproducts of RNA polymerase II, without any biological function. However, many biological functions of lncRNAs were discovered recently, conferring lncRNAs one of the most important mediators in physiological and pathological processes [20]. Generally, lncRNAs exert their roles through regulating the expression, stabilities or activities of proteins [21]. LncRNAs participate in gene expression regulation by recruiting remodeling complexes to the promoter of nearby or distant genes, and exert their roles in *cis* or in *trans*. Meanwhile, lncRNAs also interact with some key signaling molecules, and participate in the activation of signaling pathways through regulating the stabilities or activities of interaction proteins [22–24]. Although the biological roles of lncRNAs were widely investigated, their roles in liver TIC self-renewal remain unclear.

*SAMMSON* is a long noncoding RNA located on chromosome 3p13-3p14, a frequent amplified region in melanomas [25]. *SAMMSON* is a target of transcription factor SOX10 and interacts with p32 to enhance its oncogenic function [25]. *SAMMSON* recruits p32 to mitochondrial localization and silencing of *SAMMSON* disrupts mitochondrial function of melanoma cells, conferring *SAMMSON* a new target for melanoma elimination. A recent work also revealed that *SAMMSON* is required for melanoma cell viability [26]. However, the role of *SAMMSON* in liver cancer and liver TICs is unclear. Here we found high expression of *SAMMSON* in liver cancer and liver TICs. *SAMMSON* initiates Wnt/β-catenin activation and the self-renewal of liver TICs. *SAMMSON* interacts with and recruits EZH2 to the promoter of CTNNBIP1, and inhibits its transcription initiation.

The article "SAMMSON drives the self-renewal of liver tumor initiating cells through EZH2-dependent Wnt/β-catenin activation" was retracted in 2022. Reasons: duplicated images; original data or images not available.

## RESULTS

### *SAMMSON* is highly expressed in liver cancer and liver TICs

*SAMMSON* plays an essential role in melanoma cell viability and metabolic vulnerability, while, its role in liver tumorigenesis and liver TIC self-renewal is unknown. Accordingly, we detected the expression levels of *SAMMSON* in liver cancer. *SAMMSON* is highly expressed in HCC samples, especially in advanced HCC samples (Figure 1A, 1B). Interestingly, only a small subset cells showed high expression of *SAMMSON* in HCC samples, especially in early HCC samples (Figure 1B).

**Figure 1:** *SAMMSON* is highly expressed in live cancer and liver TICs **(A)** RNA were extracted from 19 peri-tumor samples, 7 early hepatocellular carcinoma (HCC) and 12 advanced HCC (aHCC) samples, followed by realtime PCR detection for *SAMMSON* expression. The average expression level of peri-tumor samples was defined as 1. **(B)** *SAMMSON* expression profiles in peri-tumor, early HCC (eHCC) and advanced HCC (aHCC). Left panels were typical images of *in situ* hybridization, right panels were statistical results. Scale bars, 50 μm. **(C)** Liver TICs were enriched from primary cells using TIC surface marker CD133, followed by *SAMMSON* detection with realtime PCR. **(D)** Liver oncospheres and non-spheres were collected for *SAMMSON* detection with realtime PCR. *SAMMSON* expression levels in non-sphere served as control. **(E)** Fluorescence *in situ* hybridization (FISH) results showed high expression of *SAMMSON* in oncospheres. c-Myc served as a positive control. Scale bars, 10 μm. **(F)** Nuclear-cytoplasmic segregation was performed and subcellular location of *SAMMSON* was detected with realtime PCR (left panels). The efficiency of nuclear-cytoplasmic segregation was detected with Western blot (right panels). Data were shown as means±s.d. ^**^P < 0.01; ^***^P < 0.001 by two-tailed Student’s t test. Data are representative of three independent experiments.

We then enriched liver TICs from HCC primary samples using TIC surface marker CD133, followed by *SAMMSON* mRNA detection. Compared with CD133^-^ non-TICs, TICs showed high *SAMMSON* expression (Figure 1C). Similarly, high expression of *SAMMSON* was also found in oncospheres (Figure 1D). We then confirmed *SAMMSON* expression profiles in oncospheres and non-spheres with fluorescence *in situ* hybridization (FISH), and found *SAMMSON* was highly expressed in spheres (Figure 1E). To our surprise, *SAMMSON* was mainly located in nucleus according to ISH and FISH data (Figure 1B, 1E), but not mitochondrial localization. Accordingly, we performed nuclear-cytoplasmic segregation and examined the subcellular location of *SAMMSON*, and once again we found the nuclear location of *SAMMSON*. Altogether, *SAMMSON* was highly expressed in liver cancer and liver TICs, with nuclear location.

The article "SAMMSON drives the self-renewal of liver tumor initiating cells through EZH2-dependent Wnt/β-catenin activation" was retracted in 2022. Reasons: duplicated images; original data or images not available.

### *SAMMSON* is required for liver TIC self-renewal

We then explored the role of *SAMMSON* in TIC self-renewal. Sphere formation assay is the most widely-accepted experimental system to detect TIC self-renewal. So we knockdown *SAMMSON* with antisense oligos (ASO), followed by sphere formation. *SAMMSON* silenced cells showed impaired sphere formation (Figure 2A). We further examined the long-term self-renewal of *SAMMSON* silenced TICs, and also found attenuate self-renewal in long-term incubation (Figure 2B). These data indicate the critical role of *SAMMSON* in liver TIC self-renewal.

**Figure 2:** *SAMMSON* is required for liver TIC self-renewal **(A)** *SAMMSON* silenced cells were established with antisense oligos (ASO) (left panels), followed by sphere formation assay. Typical photos of oncospheres were shown in middle panels and sphere initiating ratios were shown in right panels. **(B)** Sequential sphere formation assay were performed with *SAMMSON* silenced cells. 1^st^, the first passage; 2^nd^, the second passage; 3^rd^, the third passage; 4^th^, the fourth passage. **(C)** 1×10^4^ *SAMMSON* silenced and control cells were used for transwell assay, and invasive cells were visualized by crystal violet staining. **(D)** 1×10^6^ *SAMMSON* silenced and control cells were subcutaneously injected into BALB/c nude mice, and tumor weight was measured 1 month later. **(E, F)** 10, 1×10^2^, 1×10^3^, 1×10^4^, and 1×10^5^ *SAMMSON* silenced cells (ASO) and control cells (Ctrl) were subcutaneously injected into BALB/c nude mice for 3 months’ tumor formation. The ratios of tumor-free mice were shown (E). TIC ratios were calculated by Extreme Limiting Dilution Analysis (ELDA) (F). CI, Confidence interval. **(G)** *SAMMSON* overexpressed cells were established (left panels) and sphere formation assay was performed (middle and right panels). Representative images were shown in middle panels and calculated ratios were in right panels. **(H)** 1×10^4^ *SAMMSON* overexpressed and control cells were used for transwell assay, and invasive cells were visualized by crystal violet staining. **(I)** 1×10^6^ *SAMMSON* overexpressed cells (oe *SAMMSON*) and control cells (oeVec) were injected into BALB/c nude mice, and tumor weight was measured 1 month later. **(J, K)** 10, 1×10^2^, 1×10^3^, 1×10^4^, and 1×10^5^ *SAMMSON* overexpressing (oeSAMMSON) and control (oeVec) cells were subcutaneously injected into BALB/c nude mice for tumor initiation as E, F. Scale bars, A, G, 500 μm. Data were shown as means±s.d. ^**^P < 0.01; ^***^P < 0.001 by two-tailed Student’s t test. Data are representative of three independent experiments.

The article "SAMMSON drives the self-renewal of liver tumor initiating cells through EZH2-dependent Wnt/β-catenin activation" was retracted in 2022. Reasons: duplicated images; original data or images not available.

Considering the critical role of TICs in tumor propagation and initiation, we then detected tumor propagation and initiation of *SAMMSON* silenced cells. Impaired tumor invasion capacity was found upon *SAMMSON* knockdown (Figure 2C). We then subcutaneously injected 1×10^6^ cells into BALB/c nude mice, and measured tumor weight one month later. *SAMMSON* silenced cells formed much smaller tumors, indicating the critical role of *SAMMSON* in tumor propagation (Figure 2D). We also subcutaneously injected gradient diluted cells into BALB/c nude mice, and observed tumor formation three month later. *SAMMSON* depleted cells showed impaired tumor formation capacity, confirming the important role of *SAMMSON* in tumor initiation (Figure 2E, 2F).

We also established *SAMMSON* overexpressed cells, and detected self-renewal and propagation of TICs. *SAMMSON* silenced cell showed enhanced sphere formation ability (Figure 2G), invasion (Figure 2H) and propagation (Figure 2I), echoing to the silenced cells. *SAMMSON* overexpressing cells showed enhanced tumor initiation and increased TIC ratios, further confirming the critical role of *SAMMSON* in liver TICs (Figure 2J, 2K). These data confirmed the role of *SAMMSON* in liver TIC self-renewal. Taken together, *SAMMSON* drove the self-renewal of liver TICs.

### *SAMMSON* drove liver TIC self-renewal through Wnt/β-catenin signaling

We then explored the molecular mechanism of *SAMMSON* in liver TIC self-renewal. There were several signaling pathways participated in liver TIC self-renewal, including NFkB, Wnt/β-catenin signaling, Notch signaling and Hedgehog signaling. We detected the expression levels of target genes of these signaling and found decreased expression of Wnt/β-catenin signaling upon *SAMMSON* depletion, indicating that *SAMMSON* was involved in Wnt/β-catenin activation (Figure 3A). To further confirm the role of *SAMMSON* in Wnt/β-catenin signaling, we performed TOPFlash assay with *SAMMSON* silenced cells, and found attenuate TOPFlash activity, confirming the critical role of *SAMMSON* in Wnt/β-catenin activation (Figure 3B). Taking advantage of Western blot, we also detected the protein levels of c-Myc and CCND2, two Wnt/β-catenin target genes, and once again validated the participation of *SAMMSON* in Wnt/β-catenin signaling (Figure 3C). We also examined the expression levels of Wnt/β-catenin signaling target genes and further confirmed the function of *SAMMSON* in Wnt/β-catenin activation (Figure 3D).

The article "SAMMSON drives the self-renewal of liver tumor initiating cells through EZH2-dependent Wnt/β-catenin activation" was retracted in 2022. Reasons: duplicated images; original data or images not available.

**Figure 3:** *SAMMSON* drives liver TIC self-renewal through Wnt/β-catenin signaling **(A)** Heatmap of indicated gene expression in *SAMMSON* silenced cells (ASO) and control cells. Target genes of NFkB, Wnt/β-catenin, Notch and Hedgehog signaling pathways were measured using realtime PCR. **(B)** TOPFLash assay was performed using *SAMMSON* depleted and control cells. Luciferase activity in control cells served as loading control. **(C)** Western blot analysis for Wnt/β-catenin activation in *SAMMSON* silenced cells (ASO) and control cells. c-Myc and CCND2 were examined. **(D)** Heatmap of indicated gene expression in *SAMMSON* overexpressed cells (oeLnc) and control cells (oeVec). **(E)** *SAMMSON* overexpressed cells and control primary cells (oeVec) were treated with the indicated inhibitor, followed by sphere formation assay. The sphere formation ratios were shown. **(F)** c-Myc and CCND2 were rescued in *SAMMSON* silenced cells, followed by sphere formation assays. Left panels were typical photos and right panels were calculated ratios. Scale bars, 500 μm. Data were shown as means±s.d. ^**^P < 0.01; ^***^P < 0.001 by two-tailed Student’s t test. Data are representative of three independent experiments.

We found *SAMMSON* was required for liver TIC self-renewal and Wnt/β-catenin activation, and then we wanted to know whether *SAMMSON* involved in liver TIC self-renewal through Wnt/β-catenin signaling. We blocked the several signaling pathways using specific inhibitors and overexpressed *SAMMSON*, followed by sphere formation. Only in Wiki4 (Wnt/β-catenin inhibitor) treated cells, *SAMMSON* overexpression had no influence on liver TIC self-renewal, suggesting that *SAMMSON* induced liver TIC through Wnt/β-catenin signaling (Figure 3E). We also rescued the expression of Wnt/β-catenin target genes, and found rescue of Wnt/β-catenin signaling largely increased self-renewal, further confirming that *SAMMSON* influenced liver TIC self-renewal through Wnt/β-catenin signaling. Taken together, *SAMMSON* drove the activation of Wnt/β-catenin and the subsequent liver TIC self-renewal.

### *SAMMSON* interacts with EZH2

To further explore the molecular mechanism of *SAMMSON* in liver TIC self-renewal and Wnt/β-catenin activation. We performed RNA pulldown assay, identified the specific band of *SAMMSON* through Mass spectrum and found the interaction between *SAMMSON* and EZH2 (Figure 4A). We also confirmed their interaction using Western blot (Figure 4B). Then we constructed *SAMMSON* truncates and examined their interaction with EZH2. The results showed that the third region (#3) of *SAMMSON* is required for the interaction between *SAMMSON* and EZH2 (Figure 4C). We then performed RNA electrophoretic mobility shift assay (RNA EMSA), and also validated the binding between *SAMMSON* and EZH2 (Figure 4D). Meanwhile, RNA immunoprecipitation (RIP) assay showed that EZH2 can enrich *SAMMSON*, further confirming the interaction of *SAMMSON* and EZH2 (Figure 4E). Finally, we performed double FISH assay and found large extant of co-localization between *SAMMSON* and EZH2 in liver oncospheres (Figure 4F). Altogether, *SAMMSON* interacts with EZH2 in liver TICs.

The article "SAMMSON drives the self-renewal of liver tumor initiating cells through EZH2-dependent Wnt/β-catenin activation" was retracted in 2022. Reasons: duplicated images; original data or images not available.

**Figure 4:** *SAMMSON* interacts with EZH2 **(A)** Biotin labeled *SAMMSON* transcript was obtained *in vitro*, followed by incubation with cell lysate of oncospheres. The specific band of *SAMMSON* was identified as EZH2. **(B)** The interaction between *SAMMSON* and EZH2 was confirmed by RNA pulldown and Western blot. β-actin served as a loading control. **(C)** *SAMMSON* truncates were constructed (left panels) and RNA pulldown assays were performed. Western blot showed the third region (#3) of *SAMMSON* was required for its binding to EZH2. **(D)** *SAMMSON*-EZH2 interaction was confirmed by RNA EMSA. The third region of *SAMMSON* was used as probe. **(E)** RNA immunoprecipitation (RIP) was performed with EZH2 antibody or IgG control antibody, and the enriched RNA was examined for *SAMMSON* enrichment. Data were shown as means±s.d. **(F)** Double FISH of *SAMMSON* and EZH2 in oncospheres. Yellow regions denote the co-localization of *SAMMSON* and EZH2. Scale bars, 20 μm. Data are representative of three independent experiments.

### *SAMMSON* recruits EZH2 to *CTNNBIP1* promoter

To further investigate the role of *SAMMSON* in liver TIC self-renewal and Wnt/β-catenin activation. We explored the expression levels of the upstream of Wnt/β-catenin signaling, including Wnt receptors, components of APC complex, TCF/LEF complex, β-catenin and its inhibitor CTNNBIP1. We found enhanced expression of CTNNBIP1 upon *SAMMSON* depletion or EZH2 inhibition, indicating *SAMMSON* and EZH2 precipitated in Wnt/β-catenin activation through inhibiting CTNNBIP1 expression (Figure 5A). We also confirmed the role of *SAMMSON* and EZH2 in CTNNBIP1 expression with Western blot (Figure 5B).

**Figure 5:** *SAMMSON* recruits EZH2 to *CTNNBIP1* promoter **(A)** Heatmap of Wnt/β-catenin upstream genes. The expression levels of Wnt receptors, components of APC complex, TCF/LEF complex, β-catenin and its inhibitor CTNNBIP1 were detected using *SAMMSON* silenced and EZH2 inhibited cells. **(B)** CTNNBIP1 protein levels were detected with Western blot. β-actin served as a loading control. **(C)** ChIP and ChIRP assays were performed to determine the enrichment of EZH2 and *SAMMSON* on *CTNNBIP1* promoter, followed by realtime PCR. The combination of EZH2 and CTNNBIP1 was shown in upper panels and *SAMMSON* binding profiles were shown in lower panels. **(D)** EZH2 ChIP assay was performed using *SAMMSON* silenced (ASO) and control cells (Ctrl). Impaired binding of EZH2 and *CTNNBIP1* promoter was found in *SAMMSON* silenced cells. **(E, F)** ChIP assays were performed using indicated antibodies to detect the repressive histone modification levels. *SAMMSON* silenced cells (E) and EZH2 inhibited cells (F) were used for ChIP assay, and impaired repressive modification was found upon *SAMMSON* or EZH2 loss of function. Data were shown as means±s.d. ^**^P < 0.01; ^***^P < 0.001 by two-tailed Student’s t test. Data are representative of three independent experiments.

The article "SAMMSON drives the self-renewal of liver tumor initiating cells through EZH2-dependent Wnt/β-catenin activation" was retracted in 2022. Reasons: duplicated images; original data or images not available.

Considering that EZH2 is a core component of PRC2 chromatin remodeling complex, we raised a hypothesis that *SAMMSON* recruited EZH2 to CTNNBIP1 for transcription repression. To test this, we performed a ChIP assay with EZH2 antibody and ChIRP assay with *SAMMSON* probes. As expected, both EZH2 and *SAMMSON* can bind to the same region of *CTNNBIP1* promoter (Figure 5C). More importantly, attenuate interaction between EZH2 and CTNNBIP1 was found in *SAMMSON* silenced cells, indicating that *SAMMSON* recruited EZH2 to *CTNNBIP1* promoter (Figure 5D). What is more, we also determined *CTNNBIP1* promoter activity by detecting histone modification. As we know, EZH2 can inhibit transcription initiation through repressive histone modification (H3K9Me3, H4K20Me3, H3K27Me3, et, al), so we detected these modification of *CTNNBIP1* promoter. As the results indicated, both in *SAMMSON* silenced and EZH2 inhibited cells, impaired enrichment of repressive histone modification were detected, further confirming the role of *SAMMSON* and EZH2 in transcriptional repression of CTNNBIP1 (Figure 5E, 5F). Taken together, *SAMMSON* inhibits the expression of CTNNBIP1 by recruiting EZH2 to *CTNNBIP1* promoter.

### SAMMSON-EZH2-CTNNBIP1-β-catenin signaling served as targets for liver TIC elimination

We found that *SAMMSON* and EZH2 can block the expression of CTNNBIP1 to activate Wnt/β-catenin signaling. Then we further explored the role of this pathway in liver TIC self-renewal and elimination Firstly, we constructed EZH2 and CTNNBIP1 knockout cells using CRISPR/Cas9 approaches, and examined liver TIC self-renewal through sphere formation assays. *EZH2* knockout impaired liver TIC self-renewal, while, *CTNNBIP1* deficient cells showed enhanced sphere formation (Figure 6A, 6B). These results showed EZH2 and CTNNBIP1 were indeed involved in liver TIC self-renewal. Considering the inhibitory role of CTNNBIP1 in Wnt/β-catenin activation, and our discovery that EZH2 repressed CTNNBIP1 transcriptional activation, we then detected the role of EZH2 in Wnt/β-catenin activation using EZH2 inhibitors (GSK126 and GSK343). EZH2 inhibition impaired the activation of Wnt/β-catenin signaling, further confirming the regulatory of *SAMMSON* and EZH2 in CTNNBIP1 repression and Wnt/β-catenin activation (Figure 6C).

The article "SAMMSON drives the self-renewal of liver tumor initiating cells through EZH2-dependent Wnt/β-catenin activation" was retracted in 2022. Reasons: duplicated images; original data or images not available.

**Figure 6:** *SAMMSON*-EZH2-Wnt/β-catenin pathway serves as a target for liver TIC elimination **(A, B)** EZH2 and CTNNBIP1 were deleted with CRISPR/Cas9 approach (left panels), followed by sphere formation assays (middle and right). Typical images were shown in middle panels and calculated sphere formation ratios were shown in right panels. **(C)** Wnt/β-catenin activation was detected by western blot analysis with the indicated antibodies. Cells were treated with GSK126 and GSK343, two inhibitors of EZH2. **(D)** 1×10^6^ indicated treated cells were subcutaneously injected into BALB/c nude mice and tumors were obtained one month later. Tumors were weighted and scatter diagram was shown. **(E)** Immunohistochemistry of c-Myc in EZH2 and Wnt/β-catenin inhibited tumors. The indicated treated tumors were obtained and immunohistochemistry was performed using c-Myc antibody. **(F)** The indicated treated tumors were analyzed with CD133 expression profiles. CD133^+^ cells were gated and ratios were shown. Scale bars, A, B, 500 μm; E, 50 μm. Data were shown as means±s.d. ^**^P < 0.01; ^***^P < 0.001 by two-tailed Student’s t test. Data are representative of three independent experiments.

Finally, we detected the role of our discovered pathway in liver TIC propagation and liver cancer progression. We treated liver cancer with EZH2 inhibitors and Wnt/β-catenin inhibitor, followed by detection of tumor weight and severity. Both EZH2 and Wnt/β-catenin inhibitors treatment induced slower tumor propagation (Figure 6D). We also detected the proportion of liver TICs in established tumors with two TIC markers, c-Myc and CD133. Inhibitor treated tumors showed attenuate c-Myc expression (Figure 6E) and decreased CD133 proportion (Figure 6F), proving that *SAMMSON*-EZH2-Wnt/β-catenin pathway serves as a target for liver TIC elimination.

The article "SAMMSON drives the self-renewal of liver tumor initiating cells through EZH2-dependent Wnt/β-catenin activation" was retracted in 2022. Reasons: duplicated images; original data or images not available.

### Conclusions

This study explored the role of *SAMMSON* (an important lncRNA in melanoma cell) in liver cancer and liver TICs. Through interacting with EZH2 and inhibiting the transcription activation of CTNNBIP1, *SAMMSON* participates in Wnt/β-catenin activation, liver TICs self-renewal, liver cancer invasion and propagation. Additionally, we found *SAMMSON*-EZH2-Wnt/β-catenin axis served as a target for liver TIC elimination.

## DISCUSSION

Wnt/β-catenin signaling is the one of most deeply investigated pathways in TICs, especially in liver cancer and colorectal cancer [15, 27]. As we know, TICs are also termed cancer stem cells. They share many similarities to tissue progenitor cells [28]. One hypothesis for the origin of TICs is that they generate from normal tissue progenitor cells. Tissue progenitor cells accumulate more and more mutations and finally become TICs [29]. In intestine and liver, the progenitor cells show hyperactivation of Wnt/β-catenin signaling [30, 31], and correspondingly, liver cancer and colorectal cancer also show hyperactivation of Wnt/β-catenin signaling [27, 32], and so do TICs [27, 33]. Recently, more and more works explored the role of Wnt/β-catenin signaling in intestinal stem cells and colorectal TICs, while, its role in liver cancer and liver TICs is much less investigated. Here we proved that Wnt/β-catenin, accompanied with *SAMMSON* and EZH2, are involved in liver TIC self-renewal.

β-catenin is core component of Wnt/β-catenin signaling, and β-catenin stability regulation and activity regulation are precisely regulated. Upon Wnt activation, APC complex, a degrading machine of β-catenin, is disrupted [34]. β-catenin released from the APC complex translocates into nucleus and form another complex with TCF/LEF to initiate the transcription of target genes [35]. More and more modules are discovered in Wnt/β-catenin regulation, while, the role of long noncoding RNA in this process is rarely reported. Lnc β-catm promotes the interaction between β-catenin and EZH2 to enhance the methylation of β-catenin. β-catenin methylation inhibits β-catenin ubiquitinoylation and finally drives the activation of Wnt/β-catenin signaling [36]. Here, we found *SAMMSON* binds to *CTNNBIP1* promoter and recruits EZH2 to *CTNNBIP1* promoter, represses the transcription initiation of CTNNBIP1 and finally activates Wnt/β-catenin signaling. Our discovery reveals a new layer for Wnt/β-catenin regulation.

In previous report, *SAMMSON* is located on mitochondria and interacted with p38 in melanoma cells [25]; here we found *SAMMSON*’s nuclear location in liver TICs. Meanwhile, *SAMMSON* involved in mitochondrial function and viability of melanoma cells [25, 26]; here we found *SAMMSON* participates in liver TIC self-renewal. There are so many differences between our finding and previous work. In our opinion, at least two reasons account for these difference. One is the different tumor types. Liver tumor and melanoma are very different, and many regulatory networks may differ in different tumors [37]. The other one is the difference between liver cancer and liver TICs. TICs have the abilities of self-renewal, differentiation, metastasis and drug resistant, but normal tumor cells have no such characteristics [2]. Several experimental data validate that in liver TICs, *SAMMSON* is truly located in cell nucleus and interacts with EZH2.

The article "SAMMSON drives the self-renewal of liver tumor initiating cells through EZH2-dependent Wnt/β-catenin activation" was retracted in 2022. Reasons: duplicated images; original data or images not available.

EZH2 is the core component of PRC2, one of the most important chromatin remodeling complexes [38]. EZH2 methylates histone to repress transcription initiation EZH2 promotes tumorigenesis through Polycomb dependent and independent manner [39, 40]. Here we found EZH2 inhibition induced impaired liver tumor propagation and liver TIC self-renewal. As we know, tumorigenesis is a process of pathological chromatin remodeling, and many remodeling complexes showed abnormal expression levels along with tumorigenesis [41], including BRG1 [42], HDAC1/2 [43], BPTF [14]. Accordingly, inhibition of abnormal chromatin remodeling serves as an avenue for tumor targeting. Truly, several inhibitors of HDAC have been approved for clinical application [44]. Here we found EZH2 inhibitors also can eliminate liver TICs, providing a novel way for liver tumor and liver TIC targeting.

## MATERIALS AND METHODS

### Cells and samples

293T cells (ATCC CRL-3216), used for lentivirus production, were purchased from ATCC. Cells were maintained in DMEM medium, supplemented with 10% FBS (Invitrogen), 100 μg/ml penicillin, and 100 U/ml streptomycin.

Human liver cancer samples were obtained from the department of Pathology with informed consent, with the approval of the Institutional Review Board. All experiments were approved by the institutional committee of Institute of the First Affiliated Hospital of Nanchang University.

### Antibodies and reagents

Anti-histone H3 (cat. no. 4499), anti-CCND2 (cat. no. 3741), anti-EZH2 (cat. no. 5246) antibodies were from Cell Signaling Technology. Anti-β-catenin (cat. no. ab32572), anti-CTNNBIP1 (cat. no. ab129011) antibodies were obtained from Abcam. Anti-β-actin (cat. no. A1978) were obtained from Sigma-Aldrich. Phycoerythrin (PE)-conjugated CD133 (cat. no. 130098826) was purchased from MiltenyiBiotec. Anti-EEA1 (sc-53939), anti-Myc (sc-4084) antibodies were purchased from Santa Cruz Biotechnology. Alexa488-conjugated donkey anti-mouse IgG (cat. no. R37114) and Alexa594-conjugated donkey anti-rabbit IgG (cat. no. R37119) were from Molecular Probes. DAPI (cat. no. 28718-90-3) were from Sigma-Aldrich. The LightShift Chemiluminescent RNA EMSA kit (cat. no. 20158) and Chemiluminescent Nucleic Acid Detection Module (cat. no. 89880) were from Thermo Scientific. T7 RNA polymerase (cat. no. 10881767001) and Biotin RNA Labeling Mix (cat. no. 11685597910) were from Roche.

The article "SAMMSON drives the self-renewal of liver tumor initiating cells through EZH2-dependent Wnt/β-catenin activation" was retracted in 2022. Reasons: duplicated images; original data or images not available.

### TOPFlash luciferase assay

TOPFlash reporter plasmid (Addgene, 12456) and mutant FOPFlash reporter plasmid (Addgene, 12457), along with thymidine kinase (TK), were transfected into *SAMMSON* silenced cells. 36 h later, cellular luciferase activities were detected with dual-detection luciferase detection kit (cat. no. E1910, from Promega Corporation).

### Sphere formation

For sphere formation assay, 5000 primary cells were added in Ultra Low Attachment 6-well plates (Corning Company) for incubation with DMEM/F12 (Life Technologies) supplemented with B27(Life Technologies, cat. no. 17504-044), N2(Life Technologies, cat. no. 17502-048), 20 ng/ml bFGF (Millipore, cat. no. GF446-50UG) and 20 ng/ml EGF (Life Technologies, cat. no. E5036-200UG). Two weeks later, the spheres were collected and counted for sphere initiating ratios.

### Chromosome immunoprecipitation (ChIP)

We performed ChIP assays according to the manual of Upstate Biotechnology, Inc. Briefly, *SAMMSON* silenced spheres were incubated in 1% formaldehyde at 37°C for crosslinking, followed by incubation in SDS lysis buffer and subsequent ultrasonic for shearing DNA to segments of 200-1,000 bp in length. EZH2 antibody was added into samples for DNA segment enrichment.

### RNA pulldown

For RNA pulldown assays, biotin-labeled *SAMMSON* were generated *in vitro* with biotin RNA labeling mix. The labeled RNA transcript was incubated with oncospheres lysate, followed by streptavidin beads enrichment and SDS–PAGE. The interaction protein was detected with Western blot or mass spectra.

### RNA immunoprecipitation (RIP)

For RIP, liver oncospheres were incubated with 1% formaldehyde for crosslinking, and crushed with RNase-free RIPA buffer. The Supernatants were incubated with EZH2 antibody and subsequent protein A/G beads for RNA enrichment, and *SAMMSON* enrichment was examined using real-time PCR.

### Tumor proliferation and initiating assay

For tumor proliferation assay, 1×10^6^ *SAMMSON* silenced or overexpressed cells were subcutaneously injected into BALB/c nude mice for 1 month. Then tumors were obtained for weight detection. For tumor initiating assays, 10, 1×10^2^, 1×10^3^, 1×10^4^, and 1×10^5^ *SAMMSON* silenced cells were subcutaneously injected into BALB/c nude mice. Tumor initiation was observed 3 month later. For tumor propagation and initiating assay, 6-week-old BALB/c nude mice were used. For every samples, 6 mice were used.

The article "SAMMSON drives the self-renewal of liver tumor initiating cells through EZH2-dependent Wnt/β-catenin activation" was retracted in 2022. Reasons: duplicated images; original data or images not available.

### Statistical analysis

Two-tailed Student’s t tests were used for statistical analysis. P <0.05 was considered to be statistically significant.

## Abbreviation

TIC: tumor initiating cells
